# Application of Image Super-Resolution Reconstruction in Gymnastics Training by Using Internet of Things Technology

**DOI:** 10.1155/2022/8133187

**Published:** 2022-10-17

**Authors:** Sun Zhenlei

**Affiliations:** College of Physical Education, Inner Mongolia Minzu University, Tongliao 028000, China

## Abstract

Image super-resolution reconstruction, in short, is to restore some not too clear images, so that the image is more convenient to identify. It is generally used in intelligent surveillance systems and medical imaging systems in hospitals. This kind of technology is applied in many traditional algorithms. Today, the ultra-high-resolution algorithm has been revised. This paper analyzes in detail the convergence characteristics of two widely used pixel-by-pixel loss functions from theoretical and experimental perspectives, fully considers each convergence characteristic, and studies the combination of MAE and network. The MSE advantage learning method uses a single loss function to train the network. This training method can improve network performance. The level of Chinese gymnasts is relatively high, and it can even be said that they represent the most advanced level in the world. For many gymnasts, training for sharp turns is the focus of training, as well as training. Chinese gymnasts face similar problems. How to help Chinese gymnasts to improve their training quality has become a major issue in gymnastics training at this stage.

## 1. Introduction

The Internet is now the largest communication platform in society, and it plays a very important role in the collection, transmission, and storage of image information [1]. With the development of computers and the development of science and technology, professional cameras are generally accepted by people. People use scanners, smartphones, and other devices to continuously capture optical analog signals in the real world, and then capture analog digital signals to convert and calibrate images [2]. After a series of operations, save it as a digital image on the hardware device. There is no doubt that compared with the traditional binding and physical stages, digital images are easier to distribute, store, and analyze, and they become easier to understand and have greater value [3]. However, in practical applications, capturing and distributing higher resolution images are usually severely limited in hardware and software. By improving the technical level of additional metal oxide semiconductor or CCD devices in the camera to improve the resolution of the final image, this is usually related to economic development [4]. Generally, improvements are generally limited and it is impossible to achieve complete optimization. In addition, due to differences in transmission networks, the resolution of digital images is also limited. In special cases such as aerial remote sensing, medical imaging, microscopic imaging, and aerial photography, it is more difficult to obtain high-resolution images [5].

## 2. Related Work

Literature shows that people think that deep learning algorithms do not need to prespecify too much prior knowledge in comparison with traditional algorithms, and traditional algorithms are too old fashioned [6, 7]. This is a daunting task for anyone. In recent years, deep learning has become stronger in many key areas of image processing. Therefore, domestic and foreign scientists have learned lessons from the success of this technology in other fields and have proposed a method of image resolution reconstruction based on deep learning. In the literature, the idea of sparse coding method is combined. At first, we used traditional algorithm, but then we started to use SRCNN, but using SRCNN algorithm is only a recommendation [8]. Literature established a three-layer convolutional neural network, which can be trained from beginning to end [9, 10]. For the reconstruction of super-resolution images, deep learning is the most effective method. It has certain efficiency, and all of these are better than those at the time. VDSR is actually a high-resolution image reconstruction technology on the Internet. It belongs to the VG network of image classification and creates a new network system. It also has the concept of total difference, which simplifies the autonomous learning process, so it basically occupies all areas of SR. This also shows its excellence [11]. As the depth increases, the receiving range of the network becomes wider, and the network can obtain more information, which is conducive to our transformation [12]. It is proposed to use recurrent neural networks in the field of ultra-high resolution. In the literature, a cyclic residual neural network for ultra-high-resolution algorithms is proposed [13]. Compared with traditional algorithms and SRCNN algorithms, it is a resolution algorithm with integrated performance. The entire neural network area is searched, and finally information is obtained. In the literature, sub-pixels are proposed, and the convolution structure is used to replace the deconvolution structure [14]. It is proposed to calculate the similarity between the generated image and the original image in the feature space, and then PerceptualLoss function is proposed in the literature, which is applied to image transformation and can be used to train higher-order images or improve the resolution network. In addition, because of the differences in transmission networks, the resolution of digital images is also limited, such as aerial remote sensing, medical imaging, and microscopic imaging. In special cases such as aerial photography, it is more difficult to obtain high-resolution images. Literature suggests using generative adversarial networks to make the network inference results of natural images more diversified [15].

## 3. Research on Image Super-Resolution Reconstruction

### 3.1. Internet of Things Technology

#### 3.1.1. Description of the Internet

In the early years, around 1999, some scholars gave a brief overview of the concept of the Internet of Things. They explained that the Internet is actually a huge network platform composed of countless computer areas, including wireless data transmission, EPC coding, and other technologies. It can exchange global freight information in real time, which is an advanced technology used by logistics companies to exchange information and manage inventory.

#### 3.1.2. Feature Points of Internet Technology

The goal of the Internet is to monitor and track goods on a global scale and to improve the level of control over the production, storage, transportation, and sales of materials. With the development of barcode technology, this new technology can effectively improve the operational management of sales, transportation, and product tracking and optimize the inventory management process. The special features are as follows. First, the implementation of a unique object identification and barcode encoding system can only reach the classification management level. The Internet of Things EPC coding technology allows you to implement the uniqueness of a single project code and control the tracking of a single project. Second, logistics information can be monitored, and logistics information can be updated anytime and anywhere. The Internet can use RFID scanning technology to scan the EPC label on the goods, know its price and information, and facilitate our understanding. Then, information can be sent through the Internet for real-time monitoring and tracking of logistics information. Third, each inventory control connection can query product status and exchange information through Internet and RFID technology.

#### 3.1.3. The Basic Structure and Effectiveness of the Internet

The basic structure of the Internet is divided into a perception layer, a network layer, and an application layer. The basic structure and performance map of the Internet are shown in Figure 1.

RFID technology, WSN technology, EPC technology, Zigbee technology, GPS technology, and GIS technology constitute a key part of the Internet.

#### 3.1.4. RFID Technology

RFID is a non-contact automatic identification technology, based on the transmission of non-contact information and the identification of transmission information to carry out high-frequency signal spatial communication, which can contribute to the rapid development of modern logistics industry and reduce transportation and management costs. RFID technology has the following characteristics. (1) It can independently identify RFID readers and use radio waves to locate and track targets and store required information. (2) The function of adapting to the environment is extremely strong, and RFID has strong penetrating power. It can pass through opaque materials, such as wood and paper, and can transmit data over long distances. (3) The information in the reusable RFID electronic tag can be changed, deleted, and reused many times.

#### 3.1.5. WSN Technology

The WSN technology is composed of sensor units of independent network nodes. Its characteristics are (1) low power consumption; (2) low cost consumption; and (3) miniaturization. It can not only detect and monitor all the time and understand and record the environment in the network coverage area but also analyze and process information and wirelessly transmit the information to the detector.

#### 3.1.6. EPC Technology

The EPC technology is a global unified identification system developed by the United States, which assigns unique EPC codes to individual items, uses electronic tags as carriers, uses RFID technology to collect and exchange information, and uses EPC networks to transmit and store data. The main feature of the EPC technology is as follows. EPC technology can identify products on a global scale, is usually applicable to all links and nodes of inventory management, and can produce very significant effects. First of all, the EPC system is the largest open platform of the Internet. Secondly, the EPC system is highly interactive. A high degree of interactivity is the basis for collaboration between the Internet and EPC. Finally, the EPC system is flexible and sustainable, so there is no need to replace the original system when upgrading.

#### 3.1.7. Zigbee Technology

The advantage of Zigbee is that it has a short-distance, low-cost, and low-speed two-way radio communication technology, which can transmit data over a short distance with low power consumption and low transmission speed. Short-distance data transmission is its biggest feature, and the transmission rate is usually 151 to 250 kbps. Zigbee is designed with low power consumption in mind, and two AA batteries can be used for up to six months. Low performance and simple protocols can reduce costs. It is safe and reliable. Electromagnetic waves are easily affected by wireless interference. Zigbee uses IEEE802.15.4 wireless communication protocol and CSM-CA technology to resolve this conflict.

#### 3.1.8. Global Positioning System

It is a satellite navigation system developed by the U.S. Department of Defense. It has the characteristics of continuity, weather resistance, and high accuracy. It can provide global users with high-precision, low-cost, and three-dimensional information about position, speed, and accurate timing. The use of GPS has rapidly improved the level of global informatization and provided technical support for the development of the digital economy.

#### 3.1.9. Geographic Information System

It is a technical system based on computer hardware and software systems, used to collect, manage, store, calculate, analyze, describe, and display spatially consistent geographically distributed data on all or part of the Earth's surface. GIS is widely used in resource management, research, and development planning.

### 3.2. Basic Theory and Classic Algorithm of Image Super-Resolution Reconstruction

To develop ultra-high-resolution algorithms, you need to understand the basis of digital imaging theory. In addition, image super-resolution vividly shows the evolution process, and it is also important to understand how to evaluate the quality of high-resolution images. Generally, super-high-resolution problems can be divided into two types: super-high-resolution frame resolution and super-sequential frame resolution. Although the focus of this research is on SISR, this section is based on UHR and SISR algorithms with high correlation between sequences and briefly outlines the UHR domain without any difference, including image degradation models, image quality evaluation standards, and classic algorithms.

Single-frame ultra-high-resolution reconstruction usually requires reconstruction from low-resolution images into ultra-high-resolution images frame by frame. Low-resolution images are the basis of high-resolution images and can also correspond to multiple high-resolution images. Before defining the ultra-high-resolution algorithm, first define the image degradation model. The probability distribution of the degradation function and additive noise is fixed to a certain extent and can be expressed as the following formula:

(1) $$\begin{array}{c} I_{LR}=H\left(I_{HR}\right)+n_{\sigma }\text{.} \end{array}$$

Among them, ILR is the degraded low-resolution image, IHR is the original high-resolution image, and *σ* is the noise figure. Equation (2) is given with the downsampling method ↓_s_ and downsampling factor *s*:

(2) $$\begin{array}{c} I_{LR}=G_{blur}\left(I_{HR}\right){↓}_{s}+n_{\sigma }\text{.} \end{array}$$

Among them, most methods use n*σ* to represent Gaussian white noise and use bicubic interpolation to calculate the approximate Gblur value. The model of super-resolution problem in a single image is shown in Figure 2.

Regarding the definition of the model, the formula for the super-resolution rate is

(3) $$\begin{array}{c} I_{SR}=F_{S}\left(P\left(I_{LR}\right)\right)\text{.} \end{array}$$

Among them, *P* represents the preprocessing of low-resolution images, which probably includes filtering waves, reducing noise, calculating the average difference to make it normal, spatial mapping, etc., even without any operation, and *F*_*s*_ represents sampling as a super-high-resolution problem rate.

The evaluation criteria can be divided into subjective evaluation and objective evaluation. Full reference method, partial reference method, and no reference method are the three major branches of evaluation. Among them, the maximum signal-to-noise ratio and structural similarity in the complete reference method and the average opinion score in the subjective method are the most important and commonly used evaluation criteria in recent years, as well as the main evaluation criteria.

The maximum signal-to-noise ratio in signal processing is the maximum signal strength and destructive noise power that affect the accuracy of its expression. When evaluating image quality, it is expressed as a real image. Estimate the logarithm of the mean square error between the image and the maximum signal level of the image. If there is an image *X* that needs to be evaluated and a reference image with a valid *Y* value whose height and width are, respectively, *N* and *H*, the MSE expression will be

(4) $$\begin{array}{c} MSE=\frac{1}{H\times W}\overset{H}{\underset{i=1}{\sum }}\overset{W}{\underset{j=1}{\sum }}{\left(X\left(i,j\right)-Y\left(i,j\right)\right)}^{2}\text{.} \end{array}$$

MSE can calculate PSNR as follows:

(5) $$\begin{array}{c} PSNR=10\;\log_{10}\left(\frac{{\left(2^{n}-1\right)}^{2}}{MSE}\right)\text{.} \end{array}$$

The value of PSNR is inversely proportional to distortion; the larger the value, the smaller the distortion. PSNR is the most frequently used and widely used tool today. However, the human eye has a strong difference in spatial contrast, while the human eye is not so sensitive to the brightness difference. The environment affects people's eyeballs because the assessment results usually do not match people's subjective visual perception.

The spatial structure of natural images manifests itself as a strong correlation between adjacent pixels in the same image, and the important information we need can be obtained through this correlation. Assuming that the human visual system receives the image structure information, it can be judged by the brain whether it has distortion. Generally, the quality score has a great relationship with the distortion, but the image correlation of PSNR in the spatial neighborhood is of no use. Similar structure is shown in Figure 3.

The measurement of SSIM index can be composed of three parts: brightness, contrast, and structure. The details are as follows:

(6) $$\begin{array}{c} \mu_{x}=\frac{1}{N}\overset{N}{\underset{i=1}{\sum }}x_{i},\mu_{y}=\frac{1}{N}\overset{N}{\underset{i=1}{\sum }}y_{i}\text{.} \end{array}$$

The formula shown in the above formula is about the comparison function of brightness, and the estimated value is calculated by the following formula:

(7) $$\begin{array}{c} l\left(x,y\right)=\frac{2\mu_{x}\mu_{y}+C_{1}}{\mu_{x}^{2}\mu_{y}^{2}+C_{1}}\text{,} \end{array}$$

(8) is the comparison function:

(8) $$\begin{array}{c} c\left(x,y\right)=\frac{2\sigma_{x}\sigma_{y}+C_{2}}{\sigma_{x}^{2}\sigma_{y}^{2}+C_{2}}\text{.} \end{array}$$

The contrast function is estimated by contrast and brightness, and the estimated value of the structure contrast function is:

(9) $$\begin{array}{c} s\left(x,y\right)=\frac{\sigma_{xy}+C_{3}}{\sigma_{x}\sigma_{y}+C_{3}}\text{.} \end{array}$$

Due to the unstable type of *C*_1_, *C*_2_, and *C*_3_ in the formula, we usually take *C*_1_ equal to 2, *C*_2_ equal to 2, and *C*_3_ equal to *C*_2_ divided by 2. The number of bits is *n*, *L* is 2*n* − 1, *K*_1_ is equal to 0.02, and *K*_2_ is equal to 0.04. The final completeness calculation formula is as follows:

(10) $$\begin{array}{c} SSIM\left(x,y\right)=\left[l{\left(x,y\right)}^{\alpha }\right]\left[c{\left(x,y\right)}^{\beta }\right]\left[s{\left(x,y\right)}^{\gamma }\right]\text{.} \end{array}$$

The magnitude of the SSIM value is inversely proportional to the degree of distortion. Then, MSSIM is expressed as

(11) $$\begin{array}{c} MSSIM\left(X,Y\right)=\frac{1}{M}\overset{M}{\underset{i=1}{\sum }}SIMM\left(x_{i},y_{i}\right)\text{.} \end{array}$$

The opinion score is a subjective evaluation standard used to evaluate the quality of the image in the image field. As mentioned in the previous article, PSNR can measure the pixel-by-pixel error between two images, and the evaluation results can easily be inconsistent with people's subjective feelings. Therefore, Ledig and others used opinion scoring criteria for ultra-high-resolution images. The quality assessment confirmed this phenomenon, and the opinion score ratings are as follows:

(12) $$\begin{array}{c} MOS=\frac{\sum_{n=1}^{N}R_{n}}{N}\text{.} \end{array}$$

The value of MOS is usually a valid number in the range of 1–5, but the opinion score value is also affected by mathematical characteristics and distortion. For example, when evaluating objects, the gap between “good” and “normal” becomes smaller than the gap between “good” and “very good.” The gap between them is even greater, and in successive tests, subjects usually give scores across the entire list of scores. In a specific test process, different people's assessments of the same picture will be very different, the number of topics is also variable, and every time the same number of participants is sought, it is not consistent with reality. For the above reasons, the stability and efficiency of opinion scores were questioned in a clear experiment. The main topic in the field of super-resolution is the basic method of image reconstruction. This section will briefly introduce some typical classic algorithms, take a set of data for PSNR comparison, and compare visual performance.

The method based on interpolation is an idea about image restoration, which has high applicability. Therefore, in this algorithm, we compare the high-resolution image with the low-resolution image, and we find that the pixel value of the high-resolution image is based on the corresponding position of the low-resolution image.

Nearest neighbor interpolation includes assigning the value closest to the pixel to be found among the four neighboring pixels of the pixel to be found. The advantage is that this method is convenient for us to calculate and will not be so troublesome, but the disadvantage is that it will cause the gray space to be discontinuous, which will easily lead to blocking and overlap. The bilinear interpolation method is shown in Figure 4.

Bilinear interpolation is an algorithm that uses surrounding pixels to determine the interpolated pixel value. Perform linear interpolation in both directions to obtain predicted pixel values as shown in the figure. In Figure 4, four pixels *Q*_11_, *Q*_12_, *Q*_21_, and *Q*_22_ are known to form a rectangle. To estimate the value of the interpolation point *P* of the pixels within the rectangle, the pixels at the points *R*_1_ and *R*_2_ must first be determined using linear interpolation. Assuming that the pixel value of point *X* is expressed as *f* (*X*), the pixel value can be calculated according to the following formula:

(13) $$\begin{array}{c} f\left(R_{1}\right)=\frac{x_{2}-x}{x_{2}-x_{1}}f\left(Q_{11}\right)+\frac{x-x_{1}}{x_{2}-x_{2}}f\left(Q_{21}\right)\text{,}\\ f\left(R_{2}\right)=\frac{x_{2}-x}{x_{2}-x_{1}}f\left(Q_{12}\right)+\frac{x-x_{1}}{x_{2}-x_{2}}f\left(Q_{22}\right)\text{.} \end{array}$$

In the same way, we can obtain the following formula:

(14) $$\begin{array}{c} f\left(P\right)=\frac{y_{2}-y}{y_{2}-u_{1}}f\left(R_{1}\right)+\frac{y-y_{1}}{y_{2}-y_{1}}f\left(R_{2}\right)\text{.} \end{array}$$

Although the speed of bilinear interpolation is slower than that of nearest neighbor interpolation, it has great performance advantages and overcomes the effects of anti-aliasing and image blocking. However, if bilinear interpolation is used for four adjacent pixels, the slope of the resulting surface will not match the features of the partial image, so the anti-aliasing function produced by bilinear interpolation may adversely affect image details.

The bicubic interpolation technique assumes that the pixel value of any point in the same interpolation area can be calculated, as shown below:

(15) $$\begin{array}{c} \begin{array}{c} f\left(x,y\right)=\overset{3}{\underset{i=0}{\sum }}\overset{3}{\underset{j=0}{\sum }}a_{ij}x^{i}y^{j}=\left[\begin{array}{cccc} x^{3} & x^{2} & x & 1 \end{array}\right]\left[\begin{array}{cccc} a_{3,3} & a_{3,2} & a_{3,1} & a_{3,0}\\ a_{2,3} & a_{2,2} & a_{2,1} & a_{2,0}\\ a_{1,3} & a_{1,2} & a_{1,1} & a_{1,0}\\ a_{0,3} & a_{0,2} & a_{0,1} & a_{0,0} \end{array}\right]\left[\begin{array}{c} y^{3}\\ y^{2}\\ y\\ 1 \end{array}\right]\\ f\left(x,y\right)=X^{T}AY\text{.} \end{array}\text{,} \end{array}$$

It can be simplified to the following formula:

(16) $$\begin{array}{c} \left[\begin{array}{cccc} f\left(x_{0},y_{0}\right) & f\left(x_{0},y_{1}\right) & f\left(x_{0},y_{2}\right) & f\left(x_{0},y_{3}\right)\\ f\left(x_{1},y_{0}\right) & f\left(x_{1},y_{1}\right) & f\left(x_{1},y_{2}\right) & f\left(x_{1},y_{3}\right)\\ f\left(x_{2},y_{0}\right) & f\left(x_{2},y_{1}\right) & f\left(x_{2},y_{2}\right) & f\left(x_{2},y_{3}\right)\\ f\left(x_{3},y_{0}\right) & f\left(x_{3},y_{1}\right) & f\left(x_{3},y_{2}\right) & f\left(x_{3},y_{3}\right) \end{array}\right]=\left[\begin{array}{c} X_{0}^{T}\\ X_{1}^{T}\\ X_{2}^{T}\\ X_{3}^{T} \end{array}\right]A\left[\begin{array}{cccc} Y_{0} & Y_{1} & Y_{2} & Y_{3} \end{array}\right]\text{,}\\ F=X^{T}AY\text{.} \end{array}$$

The matrix *A* can be expressed as follows:

(17) $$\begin{array}{c} A={\left(X^{T}\right)}^{-1}{AY}^{-1}=\left(X^{-1}\right)AY^{-1}\text{,}\\ f\left(x,y\right)=\left[\begin{array}{cccc} x^{3} & x^{2} & x & 1 \end{array}\right]{\left(X^{-1}\right)}^{T}{AY}^{-1}{\left[\begin{array}{cccc} y^{3} & y^{2} & y & 1 \end{array}\right]}^{T}\text{.} \end{array}$$

Although this calculation method has a large amount of calculation, the accuracy of the result is higher. We generally used such methods in the early days. The comparison chart of three interpolation methods is shown in Figure 5.

The three interpolation methods have their own advantages and disadvantages. Figure 5 shows the closest neighbor in the image “baboon.png” in the dataset Set14. The four-fold upsampling pair of the bilinear and bicubic interpolation methods shows each high resolution. SSIM and PSNR indicators are used between rate images and real images. The pictures about bicubic interpolation and bilinear interpolation are very similar, but their numerical performance is quite different. In previous super-resolution studies, this was also a thorny issue, namely, the relationship between numerical performance and sensor quality.

The reconstructed image usually first models the image degradation process, and uses the degenerated prior knowledge to constrain the decision space. There are three main methods.

Iterative backprojection must first use formula (18) to create a degradation model between high-resolution and low-resolution images:

(18) $$\begin{array}{c} I_{LR}=H\left(I_{HR}\right)\text{.} \end{array}$$

Among them, high-resolution image, low-resolution image, and analog degradation function are represented by IHR, ILR, and *H*, respectively. If the existing low-resolution ILR observation image has the high-resolution image ISR estimated by the current step size, the current high-resolution image is injected into the degradation model to obtain

(19) $$\begin{array}{c} I{'}_{LR}=H\left(I_{SR}\right)\text{.} \end{array}$$

If the difference between the observed IHR of the image and the degraded ILR is less than a certain threshold, the current ISR of the high-resolution image can be regarded as a good estimate of the actual IHR of the high-resolution image; if not, the difference between the obtained ILR image and the degraded ILR is projected back to space at high resolution, and the ISR of the high-resolution image in the current iteration state is iteratively updated until the degraded image and the observed image are smaller than the ISR.  Figure 6 shows a flowchart of the iterative backprojection method.

The theory behind the iterative backprojection method is intuitive and straightforward and can better handle the edges and details of the image. However, in practical tasks, it is difficult to determine the degradation model *H*, and there is no prior knowledge such as image structure. The solution is ambiguous and unstable and may even experience convergence difficulties.

For versatility and practicability, this article focuses on the issue of super-resolution frames. Reconstruction-based methods are mainly used to reconstruct low-resolution and multiple images. Therefore, this section focuses on the performance test and comparative analysis of classic algorithms. Algorithms generally include minimum neighborhood embedding, linear neighborhood embedding, fast sparse coding, and adaptive local adjacency regression. PSNR performance comparison of traditional SISR and RGB image algorithms is shown in Table 1.

When calculating PSNR, in order to ignore the influence of edge effects, only the peak signal-to-noise ratio at the center of the image is calculated, and the edge is far away from the wide pixel *s*, where *s* is the upsampling rate of the super-pixel. The high-resolution algorithm execution and PSNR index check are done on the RGB channel. Usually, the PSNR calculated on the *Y* channel in the YCbCr color space is as follows. The test results are shown in Table 1. In the test score table, for each dataset, at each ultra-high-resolution scale, the PSNR score with the best performance is shown in bold and the sub-optimal score is highlighted. It can be concluded that in the two learning-based methods, the performance of the four algorithms is better than bicubic interpolation.

It is necessary for us to create our own SRCNN algorithm database for us to store and collect, so that the network has prior knowledge of the relationship between high-resolution and low-resolution image display. Study the potential degradation model between high-resolution and low-resolution to allow the network to extract low-resolution images, which can be used internally to reconstruct the rich information of high-resolution images. The idea of the algorithm is similar to the classic teaching method. The difference is that powerful deep learning tools replace traditional learning algorithms. The simplest and most advanced deep learning-based super-resolution method SRCNN is compared with typical traditional methods, ranging from low to high. As shown in Table 2, SRCNN outperforms all conventional methods in terms of peak signal-to-noise ratio.

The upsampler based on the convolution sub-pixel structure is used as the upscaling operation of the network feature map, and the number of parameters and the amount of calculation fully illustrate the extended nature of the structure and the structure is simple. The network can be expanded to handle multiple scale tasks at the same time. Although the performance has decreased, it has become more flexible in terms of actual usage and network storage. Under different upsampling rates, the PSNR and SSIM performance of each UHD algorithm data set is compared. The best performance is given in italics, as shown in Table 3.

The main work is to study the basic structure residual block in the residual network: the weight normalization method replaces the batch normalization method, which makes the network training independent of the data packet size and improves the performance. The speed and stability of network convergence introduce extended activation levels and channel attention mechanisms to improve network performance to a certain extent. When the network is flat or the test image is large, the asymmetry inside the image greatly increases its value.

## 4. Research on the Training of Gymnasts

### 4.1. The Influencing Factors of Gymnast's Difficulty in Turning Movement Training

In recent years, Chinese gymnastics has developed rapidly, and the overall level of athletes has also improved significantly. This is why Chinese gymnasts often win awards in various competitions. However, with the development of gymnastics, competition among athletes has become more intense, and athletes have become increasingly strict with themselves. As the key to creating a complete set of gymnastics exercises, the difficulty of rotating sports can be analyzed based on the following factors. Training technique is the biggest influence on training. The main purpose of sports training is to improve the physical fitness and flexibility of athletes and the adaptability of complex movements, so that they can perform various movements better and achieve excellent competition results. However, when training complex movements, the training environment is also very important. Secondly, if you accidentally cause injury to an athlete during training, the injury is particularly serious and may affect the athlete's life. The development of gymnastics requires coaches to have scientific teaching methods and advanced government training systems to support athletes. Before we start training, we must do warm-up exercises. Thirdly, there exist lack of communication and lack of learning experience. Effective communication between coaches and athletes is essential for training complex movements. However, as far as the current situation is concerned, there is little communication between coaches and athletes. We cannot directly control the update of technology, which leads to the fact that the focus of training is relatively backward, and the traditional training mode is adopted, and effective communication cannot be carried out. This inevitably leads to the occurrence of the problem of learning these arts, and we must deal with it in time. Athletes are affected by the competition experience and their mental state needs to be improved.

### 4.2. The Training Strategy of Gymnasts with Difficulty in Turning Movements

For gymnasts, it is very important to establish a standard training execution framework for gymnasts' complex movement training strategies. The formulation of the training syllabus in this study is mainly divided into three training phases, and targeted training is provided for different athletes to ensure that athletes can master complex rotating movements. In order to enable beginners to perform complex rotating movements, the coach must have a complete understanding of the athlete's overall level and be good at teaching the basic content of the movements. You can use multimedia devices that support motion frames. The main points and elements of the research are explained in detail, so that the athletes can form an objective understanding of the movement, thereby forming a basic understanding of the movement. Second, once they have established a basic understanding of athletes, coaches need to make full use of interdisciplinary content to establish a basic training structure, carefully optimize and define training content, and adhere to the basic principles of gradual and orderly transition from physical challenges. With the gradual development of sports, athletes are clearly aware of the structure and sports norms of sports, and finally strengthen physical exercise. Tough turns put forward strict requirements on the special qualities of athletes. Once the initial exercise detection is established, certain qualities must be strengthened to ensure exercise performance and training continuity.

The teaching technique for difficult turns must be optimized. In the learning process, specific implementations strictly follow the established learning framework. For example, first of all, we have to do some preparatory activities to warm up. For example, before performing complex exercises, you can use a barbell to exercise your arm strength. Coaches should also timely understand the needs of athletes, communicate regularly, and change training methods for them to improve training efficiency. In the second stage, the mental health and psychological quality of athletes should be taken care of. During this period of time, the athletes have actually mastered the complex rotating movement, and the coaches need to provide psychological counseling to the athletes so that they are not nervous and proud and they better master the more complex rotating movement.

In fact, the training of gymnasts' complex twisting movements is essential, but the influence of coaches on athletes is also crucial. Fitness coaches need to keep exercising by themselves, gain more experience to educate the students, change the previous training mode, add new training modes, and make the students happy. In practice, we must first master the different physical qualities of each person to adjust the training plan, so that each person can have a different plan and finally master the complex rotating movement.

## 5. Conclusion

This article briefly introduces the development history of image resolution restoration algorithms and the current research status at home and abroad, introduces the image quality degradation model of ultra-high-resolution algorithms, and the objective standards for evaluating image quality PSNR, SSIM, and subjective opinion evaluation standards. Also, through experiment comparison, the reconstruction algorithm of various pictures is briefly introduced, and the reconstruction of pictures and the training of athletes are studied in detail. The reconstruction algorithm is mainly studied, and there are many structures and loss functions. Compared with many traditional deep learning-based algorithms, they are innovative and improved, and they are in a leading position in terms of performance or parameter sets. Therefore, in gymnastics, many athletes choose a full range of gymnastics and perform heavy physical exercises, such as rotating exercises. These complex movements are the most important assessment points and the basis for many Chinese athletes to train in the actual training process. When learning complex rotational movements, the body must be stable to perform better. Because the characteristics of the complex rotation movement in gymnastics are obvious, it is necessary to learn gradually according to its characteristics and different training levels.

## Figures and Tables

**Figure 1:** The basic structure and performance map of the Internet.

**Figure 2:** Model of super-resolution problem in a single image.

**Figure 3:** Similar structure.

**Figure 4:** Bilinear interpolation method.

**Figure 5:** Comparison chart of three interpolation methods. (a) High-resolution images and terrain details. (b) Nearest neighbor interpolation images and local details. (c) Bilinear interpolation images and local details. (d) Local details of bicubic interpolation images.

**Figure 6:** IBP algorithm flow.

**Table 1:** PSNR performance comparison of traditional SISR and RGB image algorithms.

Dataset	Super-resolution scale	Bicubic	NE-LS	NE-LLE	ESC	*A*+
		PSNR (dB)	PSNR (dB)	PSNR (dB)	PSNR (dB)	PSNR (dB)
Set5	×2	32.34	34.34	34.45	34.46	35.22
Setl4	×2	29.03	30.51	30.58	30.62	31.09
Bl00	×2	28.01	29.05	29.09	29.08	29.45
Urban100	×2	25.59	27.21	27.18	27.17	27.93
D1V2K	×2	31.12	32.58	32.63	32.65	33.19
PIRM	×2	29.31	30.54	30.66	30.66	31.06
Set5	×3	29.09	30.47	30.54	30.60	31.28
Setl4	×3	26.35	27.41	27.42	27.49	27.95
Bl00	×3	25.85	26.53	26.55	26.58	26.88
Urban100	×3	23.18	24.17	24.13	24.17	24.76
D1V2K	×3	28.35	29.30	29.32	29.36	29.77
PIRM	×3	26.64	27.43	27.48	27.51	27.82
Set5	×4	27.13	28.27	28.33	28.41	29.00
Setl4	×4	24.81	25.63	25.63	25.70	26.13
Bl00	×4	24.63	25.16	25.18	25.22	25.47
Urban100	×4	21.86	22.59	22.56	22.62	23.06
D1V2K	×4	26.81	27.56	27.58	27.63	27.98
PIRM	×4	25.16	25.77	25.80	25.85	26.11

**Table 2:** Comparison of the features of traditional methods and SRCNN.

Dataset	Super-resolution scale	Bicubic PSNR (dB)	NE-LLE PSNR (dB)	*A* + PSNR (dB)	SRCNN PSNR (dB)
Set5	×2	33.66	35.77	36.54	36.66
Set14	×2	30.23	31.76	32.28	32.45
B200	×2	28.38	29.67	30.14	30.29
Set5	×3	30.39	31.84	32.59	32.75
Set14	×3	27.54	28.60	29.13	29.30
B200	×3	25.94	26.67	27.05	27.18
Set5	×4	28.42	29.61	30.28	30.49
Set14	×4	26.00	26.81	27.32	27.50
B200	×4	24.65	25.21	25.51	25.60

**Table 3:** Performance comparison of each UHD algorithm dataset

Algorithm	Scale	Set5^[^	Setl4	Bl00	Urban100	Manga109
EDSR	×2	38.11/0.9602	33.92/0.9195	*32,32*/0.9013	32.93/0.9351	*39.10/0.9773*
ES1SRN (ours)	×2	*38.14*/*0.9604*	*34.01/0.9212*	*32.32*/*0.9015*	32.87/0.9350	*39.10*/0.9772
ES1SRN + (ours)	×2	38.24 0.9614	34.06 0.9214	32.35 0.9018	33.01,0.9373	399 8/0.9780
MSSISRN (ours)	×2	38.10/0.9601	33.94/0.9197	32.20/0.9001	32.88/0.9351	38.95/0.9761
Bicubic	×3	30.39/0.8682	27.55/0.7742	27.21/0.7385	24.46/0.7349	26.95/0.8556
*A*+	×3	32.58/0.9088	29.13/0.8188	28.29/0,7835	26.03/0.7973	29.93/0.9120
SelfEx	×3	32.58/0.9093	29.16/0.8196	28.29/0.7840	26.44/0.8088	27.57/0.8210
EDSR	×3	34.65/0.9280	30.52/0.8462	29.25*/0.8093*	28.80,0.8653	34.17/0.9476
ES1SRN (ours)	×3	*34.70/0.9295*	*30.54/0.8465*	*29.26*/*0.8093*	*28.79/*0.8651	*34.15*/*0.9473*
ES1SRN + (ours)	×3	34.74/0.9299	30.57/0.8468	29.32/0.8112	29.80/*0.8652*	34.17/0.9476
MSSISRN (ours)	×3	34.12/0.9254	30.43/0.8451	29.26/0.8092	29.74/0.8648	34.12/0.9469
Bicubic	×4	28.42/0.8104	26.00/0.7027	25.96/0.6675	23.14/0.6577	24.89/0.7866
*A*+	×4	30.28/0.8603	27.32/0.7491	26.82/0.7087	24.32/0.7183	27.02/0.8548
SelfEx	×4	30.31/0.8619	27.40/0.7518	26.84/0.7106	24.79/0.7374	27.83/0.8660
EDSR	×4	32.05/0.8910	28.53/0.7804	27.57/0.7354	26.07/0.7839	29.33/0.9002
ES1SRN (ours)	×4	32.46/0.8968	28.80/*0.7876*	*27.71/0.7420*	*26.64*/*0.8033*	*31.02*/0.9148
ES1SRN + (ours)	×4	*32.47/0.8979*	*28.82/0.7876*	*27.71*/0.7419	26.60/0.8027	30.99/*0.9149*
MSSISRN (ours)	×4	32.54/0.8991	28.87/0.7890	27.79/0.7435	26.81/0.8088	31.180.9170
Bicubic	×4	32.20/0.8928	28.65/0.7827	27.65/0.7415	26.38/0.7946	30.91/0.9137
*A*+	×8	24.40/0.6580	23.10/0.5660	23.67/0.5480	20.74/0.5160	2L47/0.6500
SelfEx	×8	25.52/0.6921	23.98/0.5969	24.20/0.5678	21.37/0.5450	22.39/0.6801
SRCNN	×8	25.33/0.6900	23.76/0.5910	24.13/0.5660	21.29/0.5440	22.46/0.6950
FSRCNN	×8	20.13/0.5520	19.75/0.4820	24.21/0.5680	21.32/0.5380	22.39/0.6730
VDSR	×8	25.93/0.7240	24.26/0.6140	24.49/0.5830	21.70/0.5710	23.16/0.7250
DRCN	×8	26.15/0.7380	24.35/0.6200	24.54/0.5860	21.81/0.5810	23.39/0.7350
LapSRN	×8	26.16/0.7414	24.38/0.6199	24.58/0.5842	21.89/0.5825	23.56/0.7387
DRRN	×8	26.96/0.7762	24.91/0.6420	*24.81*/*0.5985*	22.51/0.6221	24.69/0.7841
ES1SRN (ours)	×8	*27.11*/*0.7829*	*25.02/0.6477*	24.79/0.5978	*22.65/0.6303*	*25.01/0.7945*
ES1SRN + (ours)	×8	27.22,0.7841	25.23/0.6511	24.87/0.6014	22.77/0.6320	25.09/0.7957

## Data Availability

The data used to support the findings of this study are available from the corresponding author upon request.
